The article "Anticancer, Free Radicals, and Digestive Enzyme Inhibitory Activities of Rubus sanctus Schreb Root Four Solvent Fractions" was published in 2021. Journal: Evid Based Complement Alternat Med.

# Anticancer, Free Radicals, and Digestive Enzyme Inhibitory Activities of *Rubus sanctus* Schreb Root Four Solvent Fractions

**DOI:** 10.1155/2021/6690646

**Published:** 2021-06-16

**Authors:** Nidal Jaradat, Majdi Dwikat, Johnny Amer, Mohammed Hawash, Fatima Hussein, Mohammad Qneibi, Linda Issa, Jalal Abu Asab, Haya Hallak, Diana Nael Arar, Hala Zidan Masri, Khalil Obeid, Mohammad Sharabati, Rawan Kittaneh

**Affiliations:** ^1^Department of Pharmacy, Faculty of Medicine and Health Sciences, An-Najah National University, Nablus, P.O. Box 7, State of Palestine; ^2^Department of Biomedical Sciences, Faculty of Medicine and Health Sciences, An-Najah National University, Nablus, P.O. Box. 7, State of Palestine

## Abstract

**Background:**

Humankind used herbal products as a source of medicines since they understood their therapeutic benefits from ancient times. Therefore, the current research aimed to determine the anticancer, antioxidant, and metabolic enzyme inhibitory activities of *Rubus sanctus* (RS) root four solvent fractions for the first time.

**Methods:**

The antioxidant, antilipase, and anti-*α*-amylase potentials of (RS) four solvent fractions were evaluated using standard biomedical assays. Moreover, the DNA cell cycle of liver cancer was assessed using a propidium iodide (PI) assay. At the same time, the apoptosis activity was estimated utilizing flow the cytometry method.

**Results:**

The methanol and acetone (RS) fractions showed the highest antioxidant activity with IC_50_ values of 0.078 ± 0.22 and 0.67 ± 0.25 *μ*g/ml, respectively, compared with Trolox, which has an antioxidant IC_50_ value of 2.039 ± 0.52 *μ*g/ml. Moreover, the methanol (RS) fraction has the highest anti-*α*-amylase activity with an IC_50_ value of 20.12 ± 0.34 *μ*g/ml compared with acarbose, which has an IC_50_ value of 6.565 ± 0.3 *μ*g/ml. Also, the acetone (RS) fraction revealed the highest antilipase activity with an IC_50_ value of 6.03 ± 1.23 *μ*g/ml compared with the positive control orlistat which has an IC_50_ value of 0.39 ± 0.45 *μ*g/ml. The aqueous, methanol, acetone, and hexane fractions of the (RS) roots decreased the secretion of the *α*-fetoprotein in the liver cancer cells. The acetone fraction was the most potent *α*-fetoprotein inhibitor with an average of 237 ± 12.5% compared with the average of the untreated cells, which was 4066.6 ± 202%. The hexane fraction was the most effective in diminishing apoptosis with an average of 14.5 ± 1.6%, compared with 49% ± 2 untreated cells' average. In inhibiting cell cycle progression, it was recognized that methanol fraction seems to be the most powerful amplifier of the (RS) effect, as it increased the proportion of the cells with an average of 24.5 ± 2.2%, compared with 7.4 ± 1.8% in the doxorubicin (DOX). Data indicated a decrease in cell proliferation rate by prolonging the G2-M phase and thus slowing cancer progression. Our results suggest that (RS) roots four solvent fractions have potential anticancer activity.

**Conclusion:**

The (RS) roots four solvent fractions have potential anticancer, antioxidant, antilipase, and *α*-amylase inhibitory activities. It could be a promising source for applications in the functional food, nutraceutical, and pharmaceutical industries.

## 1. Introduction

Human beings' journey on this planet has never been comfortable, and they had learned instinctively that they have to fight for their survival, and one of the most significant wars that they fought has been against diseases. Human history with diseases goes back so long that the world's oldest disease dates as far back as 600 BC, referred to as Leprosy disease, known as Hansen's disease [1, 2]. Nowadays, the fight continues against diseases of many different types, and every day, scientists work tirelessly to find a cure for those in pain. Every day, doctors from all around the world try to help patients strive to stay alive, especially those who fell victim to a vicious illness that in the 1960s it was coded “mitotic lesion” because the cancer was a too scary word to say out loud [3].

Cancer usually occurs when healthy living cells in a specific part of the body begin to grow without a restriction. Generally, cancer cells develop from normal cells due to damage to DNA. Inherited cancers can occur; this happens when the damaged DNA is inherited from the parents. However, sometimes the DNA damage may be transpired from environmental factors such as smoking, pesticides, and chemicals. Despite that, some people might think cancer is a new disease, but it is not. It dates back so far that some of the earliest evidence of human bone cancer was found in mummies in ancient Egypt around 1600 BC [4].

It is divided into different types based on where it began; all kinds of cancer disease continue to grow, divide, and redivide instead of dying and forming new abnormal cells. There are four main types of cancer, including carcinomas, which is the most common cancer type. They occur in the tissue that coats the surface of internal organs and glands, as in prostate and breast cancers; sarcomas begin in the membranes responsible for connecting and supporting the body. So, they usually happen in parts such as muscles, nerves, joints, and bone; leukemias are known as a cancer of the blood; and finally, lymphomas originate in the lymphatic system [5].

As mentioned before, cancer cells usually start at a particular part of the body; however, sometimes it continues to grow and can be migrated to other parts of the body to develop into new tumors. This process is called metastasis [6].

Cancer is the second leading cause of death in the world after cardiovascular diseases [7]. It is noted that several types and forms of cancer can affect human health, while some of them are more deadly than others, as in the case of lung, bowel, and stomach cancers, which are considered the biggest cancer killers in the world. Lung and bowel cancers are also among the most prevalent forms of cancer reported in addition to breast cancer [8].

According to scientists, some cancers are contributed to humans' lifestyle, including lung, skin, and colon cancers which have been widely increasing over the past few years. So, all the efforts are now directed at how to prevent them. The most important aspects that should be considered are the measures of primary prevention, which include teaching people about the damage of tobacco use, guiding them to healthy diets and food, and promoting health campaigns to raise knowledge about cancer [8].

Obesity is a disease determined by a measure called BMI (Body Mass Index) calculated based on weight (kg squared) and height (meter squared). A person is obese when his BMI score is between 30 and 40 and highly obese when it is above 40 [9]. The causes of obesity vary depending on one's lifestyle. It could be due to lack of exercise and physical activity, bad eating habits, or a disease such as a thyroid disorder; genetic factors also have their effect. It affects the person's appearance and health and could lead to many life-threatening diseases, such as cardiovascular and respiratory system diseases, diabetes, gout, gallstones, and cancer. Treatment includes healthy eating, regular exercise, and weight loss medicines [10].

Diabetes mellitus is a metabolic disorder of high blood sugar levels. Causes could be due to the pancreas' inability to produce insulin (the case in type I), which is most common in children and young adults and makes up about 5% to 10% of all diabetes cases. In East Asia, the rate is almost 1 new case per 100,000 in one year. On the other hand, it could be due to insulin resistance or little production by the body (the case in type II), which makes up 90% of all cases [11, 12].

Oxidative stress is an imbalance between free radicals and antioxidants in the body. The free radicals can start doing damage to fatty tissue, DNA, and proteins in the body. This damage could lead to various diseases over time, such as atherosclerosis, diabetes, inflammatory conditions, high blood pressure, heart diseases, cancer, neurodegenerative diseases, and aging. To avoid oxidative stress, one has to make sure he gets enough antioxidants in his diet, quit smoking, wear sunscreen, avoid overeating, get plenty of sleep, and do regular exercises [13].

There are many growing plants; some are considered poisonous, while others are safe to eat. Sometimes the benefit can originate from the whole plant or, in other cases, form one or more of its parts like the roots, rhizomes, leaves, fruits, stems, barks, and flowers. These particular parts are marked by including various chemical components such as volatile aromatic oils. Other components that may be used as a dietary supplement or have a pharmacological value can be used as a source for drug development; particularly today several plants derived drugs are used throughout the world [14].

Since the beginning of life, humans have depended on nature as a source of food and medicine; people knew the importance of plants and the massive benefits they contain. To this day, researchers are astonished by the amount of scientific data obtained from plants worldwide, such as the plant's case that this study revolves on [15]. This plant is distributed in the Mediterranean, Caucasus, Black Sea, Western, and Central Asia [16]. It is called “Holy Bramble,” also known as *Rubus sanctus* Schreb (RS), and belongs to the Rosaceae family [17]. The flowering plant period is from May to September, and it is two meters high; the color of flowers is light pink and sometimes white [18], the leaves are palmate, and their underneath is very hairy. The fruits are black, juicy droplets and usually edible in many regions [19].

The leaves and roots are characterized by containing several chemical constituents such as tannins, caffeoyl sugar esters, terpenoids, and flavonoids [20]. Extracts of the (RS) aerial parts were used in folk medicine for many years, healing wounds, infected insect bites, and pimples [21]. In recent years, it was proved that herbal tea made from plant roots is used to treat rheumatism and relieve pain [21]. It was also confirmed that extracts from the leaves and roots had antimicrobial effects in treating ailments such as diarrhea [20].

To the best of our knowledge, no previous studies were established on (RS) plant roots. Therefore, the current study aims to estimate anticancer, antioxidant, and metabolic enzyme inhibitory of (RS) root four solvent fractions.

## 2. Material and Methods

### 2.1. Plant Materials

The roots of the (RS) plant were collected from the mountains of Jerusalem of Palestine in November 2018. The taxonomical characterizations and the voucher specimen code (Pharm-PCT-2065) were carried out at the Pharmacognosy Laboratory of An-Najah National University. The cleaned roots were first dried at ordinary conditions, and then an air-drying oven was used for five days with a regulated temperature (25 ± 2°C) and fixed humidity (55 ± 5 RH). Later on, the dried roots were powdered coarsely and kept in unique glassware at room temperature for future use.

### 2.2. Equipment

Microplate reader (Unilab, 6000, Mandaluyong, USA), CO_2_ incubator (Esco, 2012-74317, Changi, Singapore), inverted microscope (MRC, IX73, Hong Kong, China), UV-Visible spectrophotometer (Jenway 7315, Staffordshire, UK), vortex (Heidolph Company, 090626691, Schwabach, Germany), ultrasonic cleaner (MRC Laboratory Equipment, 1108142200049, Haifa), autoclave (MRC Laboratory Equipment, A13182, Haifa), water bath (Lab Tech, 2011051806, S. Korea), stir-mixer (Tuttnaver, 300303159, China), cooled incubator (Gallenkamp, SG92/01/244, Loc, United Kingdom), micropipette (MRC Laboratory Equipment, MPC-1000, Haifa), multichannel micropipette (MRC Laboratory Equipment, MPC-8-50, Haifa), filter papers (Whatman no. 1, USA), shaker device (Memmert shaking incubator, Germany), rotatory evaporator (Heidolph vv2000 Heidolph OB2000, Germany), grinder (Molineux model, Uno, China), balance (Red wag, AS 220/c/2, Poland), flow cytometer (Becton-Dickinson LSR II, Immunofluorimetry systems, Mountain View, CA), and freeze dryer (Millrock Technology BT85, China) were used.

### 2.3. Chemicals and Reagents

The following chemicals and reagents were used: methanol, *n*-hexane, and acetone (Lobachemie, India), DPPH (2,2-diphenyl-1-picrylhydrazyl) (Sigma-Aldrich, Germany), DMSO (dimethyl sulfoxide) (Riedeldehan, Germany), Trolox ((s)-(-)-6 hydroxy-2, 5, 7, 8-tetramethychroman-2-carboxylic acid) (Sigma-Aldrich, Denmark), *α*-amylase (Sigma, Mumbai, India), DNSA (3, 5-dinitrosalicylic acid), acarbose and doxorubicin (DOX) (Sigma, St. Louis, USA), p-nitrophenyl butyrate, orlistat, Tris-HCl buffer, and porcine pancreatic lipase type (Sigma, USA), *p-*nitrophenyl butyrate (PNPB) (Sigma-Aldrich, Schnelldorf, Germany), porcine pancreatic lipase (Sigma, MO, USA), RPMI-1640 medium (Sigma, RO883-6X, Germany), penicillin (Sigma, 03-031-113, USA), 1% streptomycin and 1% l-glutamine (Sigma, G7513, France), 10% fetal bovine serum (Sigma, 10733056001, Germany), Dulbecco's phosphate-buffered saline (DPBS) (Sigma, 79383, USA), bovine albumin (Biological Industries, Israel), and annexin-V conjugated to FITC (R&D Systems, Minneapolis, MN, USA).

### 2.4. Successive Solvent Fractionation Method

The powdered roots (75 g) were soaked in 500 ml of four solvents with various degrees of polarities. Briefly, (RS) root powder was fractionated sequentially by adding solvents of increasing polarity: first it was soaked in 500 ml of hexane (nonpolar solvent) and was placed in a shaker device at 25°C for two days, and then a suction filtration was used which worked by vacuum pressure to filtrate the mixture. The remaining (RS) plant residue was soaked sequentially in acetone (polar aprotic solvent), methanol (polar protic solvent), and water (polar protic solvent). Each of the obtained hexane, acetone, and methanol fractions were separately left in the rotavap to decrease the fractions' volume, and then each fraction was dried in the incubator. In comparison, the aqueous fraction was dried in freeze-drier apparatus. The four dried fractions were stored in the refrigerator at 4–6°C for further use [22, 23].

### 2.5. Free Radical Scavenging Assay

Methanolic stock solution (1 mg/ml) was set for (RS) roots fraction and for vitamin E analog (Trolox), which was utilized as a positive control with potent antioxidant activity. Then, various concentrations from the previous stock solution were prepared. Plant working solution (1 ml) was mixed with 1 ml freshly prepared DPPH (0.002 g/ml) methanolic solution, and 1 ml methanol was then added to the previous mixture. The blank solution contained DPPH and methanol only in a ratio of 1 : 1. The solutions were incubated at room temperature (25°C) in a dark place for 30 min. Then, their optical densities were measured by the UV/Vis spectrophotometer at 517 nm [24].

Antioxidant activity was calculated per the following equation:

(1) $$\begin{array}{c} \text{DPPH inhibition}\%=\;\frac{A_{b}-A_{s}}{A_{b}}\times 100, \end{array}$$

where *A*_*b*_ is the recorded absorbance of the blank solution and *A*_*S*_ is the recorded absorbance of the sample solution or control [25].

### 2.6. *α*-Amylase Inhibitory Activity

The *α*-amylase inhibitory activity of (RS) roots fractions was carried out according to the standard method described in [26] with minor modification. Briefly, each plant fraction was dissolved in few milliliters of 10% DMSO and then further dissolved in a buffer ((Na_2_HPO_4_/NaH_2_PO_4_ (0.02 M), NaCl (0.006 M) at pH 6.9) to give concentrations of 1000 *μ*g/ml and the following dilutions were prepared (10, 50, 70, 100, and 500 *μ*g/ml). A volume of 0.2 ml of porcine pancreatic *α*-amylase enzyme solution with a concentration of (2 units/ml) was mixed with 0.2 ml of each plant fraction and then incubated for 10 min at 30°C. After that, a 0.2 ml freshly prepared starch solution (1%) was added, and the mixture was incubated for at least 3 min. The reaction was stopped by adding 0.2 ml dinitrosalicylic acid (DNSA), and then the mixture was diluted with 5 ml of distilled water and heated for 10 min in a water bath at 90°C. The mixture was left to cool down to room temperature, and then the absorbance was taken at 540 nm. A blank was prepared following the same procedure replacing the plant fraction with 0.2 ml of the previous buffer.

Acarbose was used as a positive control following the same procedure. The *α*-amylase inhibitory activity was calculated using the following equation:

(2) $$\begin{array}{c} \alpha -\text{amylase inhibition}\%=\frac{A_{b}-A_{s}}{A_{b}}\times 100, \end{array}$$

where *A*_*b*_ is the absorbance of blank and *A*_*S*_ is the absorbance of tested sample or control [27].

### 2.7. Porcine Pancreatic Lipase Enzyme Inhibitory Method

A plant extract solution (1 mg/ml) was made by dissolving 100 mg of each plant fraction in 100 ml of 10% DMSO, and then the produced solution was diluted to obtain different concentrations (5, 25, 50, 100, 200, 300, and 400 *μ*g/ml). A lipase enzyme stock solution (1 mg/ml) was also directly prepared before use by dissolving 25 mg of lipase enzyme powder in 25 ml of 10% DMSO, and then p-nitrophenyl butyrate (PNPB) stock solution was prepared by dissolving 20.9 mg PNPB in 2 ml of acetonitrile. Then, 0.2 ml from each plant fraction prepared serial dilutions was mixed with 0.1 ml of lipase enzyme stock solution and completed with a Tris-HCl solution to reach 1 ml of volume. Then it was incubated for 15 min at 37°C in a water bath, and after 15 min 100 *μ*l of *P*NPB solution was added and incubated for 30 min at 37°C. The blank solution was prepared by mixing 100 *μ*l of lipase enzyme (1 mg/ml) with Tris-HCl solution up to 1 ml. Orlistat was used as a reference and followed the same previous steps as plant fractions. The absorbance was measured utilizing a spectrophotometer at 405 nm. However, the lipase enzyme inhibitory potential was measured using the following equation:

(3) $$\begin{array}{c} I\left(\%\right)=\frac{\left[{\text{ABS}}_{\text{blank}}-{\text{ABS}}_{\text{test}}\right]}{\left[{\text{ABS}}_{\text{blank}}\right]}*100\%, \end{array}$$

where *I* (%) is the percentage inhibition of lipase enzyme [28].

### 2.8. Cytotoxic Activity

#### 2.8.1. Cell Line

The dilution of (RS) roots extracts was done with the aqueous, methanol, acetone, and hexane solvents. Preserved extracts of 1 mg from each solvent were taken to obtain a concentration of 0.1 mg/ml. Three preparations at a final concentration of 10 *μ*g/ml of each of the stated materials were made in a total of twelve fractions. All preparations were packaged in suitable, locked containers and were sent to Hadassah Hospital Laboratories for further research. Cytotoxicity evaluation was carried out using the Hep3B cell line; cells isolated from a Japanese person's liver with liver cancer and hepatitis B have the same genotype, phenotype, and features. Hep3B is liver cancer cells characterized by the secretion of *α*-fetoprotein that is considered a tumor marker. Hep3B condition was accomplished using RPMI-1640 medium enhanced with 1% penicillin, 1% streptomycin, 1% L-glutamine, and 10% fetal bovine serum; it was adapted to pH 7.2 by Dulbecco's phosphate-buffered saline (DPBS). The cells' growing process was performed at 37°C in an ESCO cell-culture incubator, a humidified atmosphere of 95% air and 5% CO_2_ at 37°C.

#### 2.8.2. Flow Cytometry Analysis

Following cultures, the harvested Hep3B cells' adjustment to 10^6^/ml in staining buffer (in saline consisting of 1% bovine albumin was achieved. For viability measurements and apoptosis, the staining of fragmented DNA by propidium iodide (PI) and phosphatidylserine staining using annexin-V conjugated to FITC was done according to the instructions of the manufacturer. Early apoptosis was defined as annexin-V (+) but propidium iodide (-), late apoptosis was defined as annexin-V (+) but propidium iodide (+) while necrosis was defined as annexin-V (-) but propidium iodide (+). On the other hand, viable cells were defined as annexin-V (-) but propidium iodide (-). Unstained controls were used in each of the experiments, such as IgG isotype controls and FMO controls. The analysis of the cell cycle by quantization of DNA content was achieved by employing propidium iodide. The Hep3B cells' fixation was performed in cold 70% ethanol at 4°C for at least 30 min. After that, the cells were washed 2x in PBS. It was calibrated to spin at 2000 rpm to dispose of the supernatant. To ensure that only DNA was stained, the treatment of cells with ribonuclease (50 *μ*l of 100 *μ*g/ml RNase) was done. Then, cells were stained with 5 *μ*l of 50 *μ*g propidium iodide/100 ml and were analyzed using the flow cytometer (Becton-Dickinson LSR II, Immunofluorometry systems, Mountain View, CA) [29].

### 2.9. Statistical Analysis

Statistical differences were analyzed with either the 2-tailed unpaired Student's *t*-test (For comparison between two groups) or one-way analysis of variance (one-way ANOVA with Newman–Keuls' posttests among multiple groups) using GraphPad Prism 5.0. Data are shown as means ± SEM.

## 3. Results and Discussion

Throughout history, people have been struck by several diseases, that some even shaped human history like the Black Death: Bubonic Plague, which spread across Europe during the fourteenth century killing 75–200 million people, and Malaria, which claimed the lives of 200 million people in the nineteenth century alone [30, 31]. Nevertheless, as life continued, human civilization proceeded to get more advanced in the medical field that they have changed many ideas that were conceived about diseases; from this point, they were able to eradicate diseases that were once a nightmare for humanity like the case of Smallpox whose yearly death rate in the 1800s was 400,000 [32]. Plants are a natural source of many bioactive compounds. Some plants exhibit a wide range of bioactivities due to the production of secondary metabolites they produce. Such metabolites are usually produced to protect the plants from the harsh environment and natural enemies.

### 3.1. Enzyme's Inhibition Assays

Antioxidants are the substrates that prevent molecules from oxidation inside the living cells and the presence of excess oxygen species that develop lethal diseases such as cancer, Alzheimer's, atherosclerosis, and diabetes mellitus [33].

Figure 1 shows that the (RS) roots four solvent fractions have strong antioxidant activity. The (RS) methanol fraction has the highest antioxidant activity with an IC_50_ value of 0.078 ± 0.22 *μ*g/ml, which is better than the IC_50_ value of the reference antioxidant compound Trolox (Table 1), which has an IC_50_ value of 2.039 ± 0.52 *μ*g/ml. The second fraction, which has strong antioxidant potential, was the acetone fraction, an antioxidant IC_50_ value of 0.67 ± 0.25 *μ*g/ml followed by hexane and aqueous fractions.

A study conducted by Serteser et al. found that (RS) methanolic fruit extract has free radical scavenging activity with IC_50_ values of 1320 *μ*g/ml [34].

Moreover, an investigation conducted by Zengin et al. found that (RS) leaf ethyl acetate, methanol, and aqueous extracts have a free radical scavenging property with Trolox equivalent values of 24.12 ± 0.81, 347.61 ± 13.21, and 386.39 ± 10.97 mg TE/g extract, respectively [35]. Also, a study established by Jamous et al. found the ethanol extract of (RS) leaves antioxidant activity with an IC_50_ value of 0.4 ± 0.16 mg/ml [36].

Additionally, an investigation conducted on *Rubus discolor* leaf aqueous, methanol, ethanol, and acetone extracts by Veličković et al. found that the leaves have antioxidant potential with IC_50_ values of 17.31 ± 0.11, 22.46 ± 0.09, 26.54 ± 0.25 and 29.46 ± 0.80 *μ*g/ml, respectively [37].

### 3.2. *α*-Amylase Inhibitory Activity

One of the methods to lower postprandial hyperglycemia, one of the leading clinical goals to control blood glucose levels in diabetic patients, is to reduce glucose absorption in the gastrointestinal tract by repressing the enzymes responsible for the hydrolysis of carbohydrates, such as pancreatic *α*-amylase, which cleaves the *α-*(1–4) glycosidic bond of amylum yield maltotriose, maltose, and glucose [38].

Table 1 reveals that the (RS) root methanol, aqueous, acetone, and hexane fraction have potential *α*-amylase inhibitory activity with IC_50_ range of 20.12–50.9 *μ*g/ml, in comparison with acarbose, which has *α*-amylase inhibitory activity and IC_50_ value of 6.56 *μ*g/ml, the most active fraction against this enzyme was methanol fraction with IC_50_ 20.12 *μ*g/ml, as shown in Figure 2. The inhibitory activity of the fractions in compression with the positive control was presented in various concentrations. This compound is utilized in the pharmaceutical practice as a commercial drug to control postprandial hyperglycemia. Our obtained (RS) extracts have potential *α*-amylase inhibitory activity almost identical as acarbose [24].

A study conducted by Zengin et al. found that the leaf (RS) ethyl acetate, methanol, and aqueous extracts have *α*-amylase inhibitory activity with acarbose equivalent values of 0.73 ± 0.05, 0.72 ± 0.01, and 0.12 ± 0.01 mmol ACAE/g extract [35].

### 3.3. Porcine Pancreatic Lipase Inhibitory Activity

Lipase is one of the essential metabolic enzymes that endorse the hydrolysis of lipids to free fatty acids and glycerol. For that, the inactivation of lipase is one of the main goals in the pharmaceutical practice to treat overweight, obesity, hypertriglyceridemia, and hypercholesterolemia. About 60% of total dietary fat hydrolysis was established by the pancreatic lipase enzyme [28]. Thus, developing hypolipidemic agents is considered the ideal therapeutic approach to treat overweight, obesity, and other related diseases [39].

In fact, (RS) root methanol, aqueous, hexane, and acetone fractions inhibited potentially the porcine pancreatic lipase with IC_50_ values range 6.03–10.31 *μ*g/ml, and the most active fraction was acetone fraction with IC_50_ value 6.03 *μ*g/ml in comparison with the commercial antilipase drug (orlistat), which has lipase inhibitory activity with an IC_50_ value of 0.39 *μ*g/ml as depicted in Table 1 and Figure 3.

A study established by Jamous et al. found that the ethanol extract of (RS) leaves inhibited the porcine pancreatic enzyme with an IC_50_ dose of 88.1 ± 4.6 mg/ml [36].

### 3.4. Cytotoxicity

#### 3.4.1. *Rubus sanctus* Root Four Solvent Fractions Inhibit DNA Cell Cycle of Hep3B Cells

One of the current study aims was to detect whether (RS) affects cell cycle disturbances in liver cancer cells. As a result, propidium iodide-stained nuclei cells were assessed through flow cytometry analyses. Parameters of cell cycles were investigated for (RS) roots fractionated with (10 *μ*g/ml) aqueous, methanol, acetone, and hexane. The incubation of these fractions of the (RS) roots with Hep3B cells was achieved 48 h. Doxorubicin (DOX) is an anticancer drug known to inhibit cell proliferation, and DNA arrest was used as a control. Following treatment with the mentioned fractions, a significant reduction in the proportion of cells in the G1 phase, where DNA synthesis usually transpires, was noticed, as demonstrated in Figure 4. Averages of 52.5 ± 3.3%, 41.6 ± 1.5%, 56 ± 5.56%, and 50 ± 6.55% were obtained in the G1 phase following treatment with aqueous, methanol, acetone, and hexane plant fractions, respectively, as compared to 65.33 ± 1.5% obtained in DOX. There were no significant differences between the methanol fraction and each one of the declared fractions (aqueous, acetone, and hexane), respectively (*P* value < 0.05).

Also, a slight decrease of cells in the S phase, which is in charge of DNA replication, was seen after the processing of the different fractions of the (RS) roots with averages of 12.1 ± 0.8%, 11.8 ± 2.5%, 10.3 ± 1.5%, and 12.6 ± 2.08% for the aqueous, methanol, acetone, and hexane fractions respectively, compared to the average of the DOX which was 17.6 ± 0.57%; Figure 4. Moreover, the *P* value was not significant between the different fractions of the (RS) roots.

Cells proportion in the G2/M phase, in which mitosis commonly takes effect, was increased as the averages obtained after treatment of the aqueous, methanol, acetone, and hexane fractions were 10.1 ± 2.2%, 24.5 ± 2.2%, 6.9 ± 1.6, and 19.6 ± 3.0% respectively, compared to 7.4% ± 1.8 in the DOX (*P* < 0.05). No notable difference between all fractions was observed (Figure 4).

These results show that (RS) roots fractions had effects on the cell cycle of the Hep3B cells. As it was noticed, methanol fraction seems to be the most potent inhibitor since it decreased the cell proliferation rate by prolonging the G2-M phase in a time-dependent process, thus slowing cancer progression. In conclusion, these data might imply that (RS) root extracts have anticancer properties.

#### 3.4.2. *Rubus sanctus* Roots Promote Cell Death by Apoptosis

The next question was whether the aqueous, methanol, acetone, and hexane fractions of the (RS) roots that disturb the DNA content could provoke programmed cell death known as apoptosis. To investigate that, it was acknowledged that cells going through apoptosis have their phatidylserine (PS) phospholipid moved from the plasma membrane's inner face to the cell surface; hence identifying apoptotic cells can be managed by the presence of PS on the cell surface. As stated in materials and methods, the staining of PS with a fluorescent conjugate of annexin-V, a protein that is known to have a high affinity for PS, was done. The detection of the PS can be accomplished; after that, flow cytometry analysis was performed. Also, cells were stained with propidium-iodide (PI), capable of entering the cell only when the plasma membrane is impaired. Early apoptosis was appraised by positive for PS, however negative for PI. Nevertheless, it was specified from the late apoptotic and necrotic cells phase, positive for PS and PI.

Figure 5(a) demonstrates that the untreated cells (Hep3B cells alone), considered the control cells, maintain a baseline apoptotic cell population of 49%. It also represents that those cells receiving treatment from aqueous, methanol, acetone, and hexane fractions of the (RS) roots had a baseline apoptotic cell population of 55.6 ± 6.6%, 49.3 ± 3.6%, 18.2% ± 2.7, and 14.5 ± 4.2%, respectively. Hexane fraction had diminished apoptosis compared to that of the untreated cells. Moreover, the population of the late apoptotic/necrotic cells showed to increase in all the different fractions of the (RS) roots to 28.8 ± 4.4%, 37 ± 5.8%, 69.6 ± 9.6%, 67.6 ± 7.5% for the aqueous, methanol, acetone, and hexane fractions, respectively, compared to 19.6 ± 2.3% in the untreated cells. Taken together, the provided data suggest that RS extracts, while decreased necrosis of Hep3B (reductions in % annexin-V-/PI+) they shifted the cells to late apoptosis and/or early death stages through increasing % of annexin-V+/PI + indicating their effects in delaying cell death and programing them to apoptosis (*P* < 0.05).

Figure 5(b) illustrates the averages of treatment of Hep3B cells with the different fractions of the (RS) roots. Generally, the given data propose that the (RS) roots shift the cells to necrosis by prolonging the G2-M phase of the Hep3B cell cycle in a time-dependent process, which means that the (RS) roots might have anticancer potential (*P* value < 0.05).

#### 3.4.3. *Rubus sanctus* Roots Decrease *α*-Fetoprotein (AFP) Secretion from Hep3B Cells

AFP is a tumor marker and protein synthesized in the fetal liver and has been speculated to be the fetal analog of serum albumin. High AFP levels might hint at different types of cancers, such as liver cancer. Averages of the AFP's secretion from the Hep3B cells alone or under treatment from the different fractions of the (RS) roots are demonstrated in Figure 6. As noticed, the averages of AFP declined from 1205 ± 101 ng/ml in the Hep3B cells to 355 ± 30.8, 530.6 ± 43.1, 237 ± 12.5, and 268 ± 7.8 ng/ml after processing with water, methanol, acetone, and hexane treatments, respectively, with the acetone fraction being the most potent inhibitor of *α*-fetoprotein secretion (*P* value < 0.05). All of this might indicate the possibility of morphological change in the cells.

A study conducted by Selmi et al. found that the cytological analysis showed a decline in the mitotic indices in the treated (RS) roots compared with their corresponding controls at all concentrations and durations tested. This notable decrease was time- and concentration-dependent. The toxic influence of *Rubus sanctus* aqueous-alcoholic extract was identified after it was treated for 12 h with 5 mg·ml^−1^ and 10 mg·ml^−1^, while the inhibition of cell division was achieved entirely [40].

No previous studies were conducted on the roots of the (RS) plant to the best of our knowledge, and our obtained results were distinguished from previously conducted results on other (RS) parts used. These facts suggest that the (RS) roots four extracts could be used as a potential antioxidant, anti-*α*-amylase, and antilipase drug. The *Rubus sanctus* roots fractions proved their ability to cause disturbances in the cell cycle progression, primarily through the G2-M phase prolongation and decreasing apoptosis. In the case of hexane fraction and shifting cells to necrosis, it might indicate anticancer attributes in a time-dependent process.

## 4. Conclusion

The obtained results showed that the (RS) plant roots have potential antioxidant, antilipase, and anti-*α*-amylase activities. In addition, the *Rubus sanctus* root extracts decreased the tumor marker *α*-fetoprotein secretion by reducing cell proportion in both G1 and S phases and inducing prolongation of the G2-M phase. They also caused the initiation of programmed cell death by apoptosis and promoted many cells in the late apoptotic/necrotic stages. All of these processes were time-dependent, and they emphasize anticancer characteristics. Further *in vitro* and *in vivo* evaluations are required to identify the exact mechanism of action of these plant extracts and identify *Rubus sanctus* roots constituents that exhibit all these pharmacological activities. In conclusion, it could be suggested that *Rubus sanctus* root four solvent fractions may be used as a promising source for functional food, nutraceutical, and pharmaceutical application industries for the treatment and prevention of global health problems including cancer, diabetes, oxidative stress, and obesity.

## Figures and Tables

**Figure 1:** DPPH free radical scavenging property by *Rubus sanctus* roots four solvent fractions and Trolox.

**Figure 2:** *α*-Amylase inhibitory activity of *Rubus sanctus* root four solvent fractions and acarbose.

**Figure 3:** Porcine pancreatic lipase inhibitory activity by *Rubus sanctus* root four solvent fractions and orlistat.

**Figure 4:** The proportion of cells in the G1, S, and G2-M phases after processing the different fractions of the *Rubus sanctus* roots.

**Figure 5:** (a) The apoptotic cell population and the late apoptotic/necrotic cells' population alone and under treatment form the different fractions of the *Rubus sanctus* roots. (b) The percent of Hep3B cells treated with the different fractions of the *Rubus sanctus* roots (10 *μ*g/ml).

**Figure 6:** Averages of the AFP's secretion from the Hep3B cells alone or under treatment form the different fractions of the *Rubus sanctus* roots.

**Table 1:** the IC_50_ values of the evaluated fractions of *Rubus sanctus* against various enzymes.

IC_50_ (*μ*g/ml)					
Enzymes	Hexane	Acetone	Methanol	Aqueous	+ve controls
DPPH	4.71 ± 0.28	0.67 ± 0.25	0.078 ± 0.22	6.55 ± 0.23	2.04 ± 0.52^a^
*α*-Amylase	50.90 ± 1.23	29.11 ± 0.39	20.12 ± 0.34	26.90 ± 0.19	6.56 ± 0.3^b^
Lipase	8.33 ± 0.30	6.03 ± 1.23	6.51 ± 1.01	10.31 ± 0.67	0.39 ± 0.45^c^

^a^Trolox; ^b^acarbose; ^c^orlistat.

## Data Availability

The data used to support the findings of this study are available from the corresponding author upon request.
